The article "Panepoxydone Targets NF-kB and FOXM1 to Inhibit Proliferation, Induce Apoptosis and Reverse Epithelial to Mesenchymal Transition in Breast Cancer" was retracted in 2023. Reasons: duplicated images; overlap with earlier publications; unreliable data; concerns about the images.

# Panepoxydone Targets NF-kB and FOXM1 to Inhibit Proliferation, Induce Apoptosis and Reverse Epithelial to Mesenchymal Transition in Breast Cancer

**DOI:** 10.1371/journal.pone.0098370

**Published:** 2014-06-04

**Authors:** Ritu Arora, Clayton Yates, Bernard D. Gary, Steven McClellan, Ming Tan, Yaguang Xi, Eddie Reed, Gary A. Piazza, Laurie B. Owen, Windy Dean-Colomb

**Affiliations:** 1 Department of Oncologic Sciences, Mitchell Cancer Institute, University of South Alabama, Mobile, Alabama, United States of America; 2 Department of Biology and Center for Cancer Research, Tuskegee University, Tuskegee, Alabama, United States of America; University of Alabama at Birmingham, United States of America

## Abstract

**Background:**

Triple-negative breast cancer (TNBC) is a highly diverse group that is associated with an aggressive phenotype. Its treatment has been challenging due to its heterogeneity and absence of well-defined molecular targets. Thus, there is an urgent need to identify novel agents with therapeutic application. NF-κB is over-expressed in many breast cancers; thus, inactivation of the NF-κB pathway could serve as a therapeutic target. Here we report for the first time the anti-tumor activity of panepoxydone (PP), a NF-κB inhibitor isolated from an edible mushroom, in several breast cancer cell lines.

**Methods:**

We investigated the effects of PP on cell growth, migration-invasion, apoptosis and EMT-related proteins expression in MCF-7 and TNBC cell lines MDA-MB-231, MDA-MB-468 and MDA-MB-453.

**Results:**

Significant antitumor activity was seen in all cell lines, with differential responses noted in cell-line specific manner. Treatment with PP resulted in significant cytotoxicity, decreased invasion, migration and increased apoptosis in all cell lines tested. Up-regulation of Bax and cleaved PARP and down-regulation of Bcl-2, survivin, cyclin D1 and caspase 3 were noted in PP-treated breast cancer cells. The antitumor effect of PP appeared related to its ability to inhibit the phosphorylation of inhibitor of NF-κB (IκBα) with cytoplasmic accumulation. PP treatment also down-regulated FOXM1 which resulted in a reversal of EMT. Similar results were obtained after silencing of NF-kB and FOXM1.

**Conclusion:**

Altogether, these studies show, for the first time the antitumor activity of PP against breast cancer cells, in particular TNBC cells. Furthermore, it highlights the concept that optimal treatment of TNBC warrants attention to the differential sensitivity of various TNBC subtypes to therapeutic agents. These results suggest that the PP may be a potentially effective chemopreventive or therapeutic agent against breast cancer. However, additional studies are required to more fully elucidate the mechanism of antitumor effect of PP.

## Introduction

Breast cancer is one of the most common malignancies in women worldwide and the second leading cause of cancer-related mortality in women. According to the latest cancer statistics report, it was estimated that about 235,030 new cases of breast cancer would be diagnosed in 2014 and 40,430 deaths would occur [1].

Triple-negative breast cancer (TNBC) is one of the most aggressive forms of breast cancer. It is typically characterized as a morphologically high grade tumor demonstrating lack of expression of estrogen (ER), progesterone (PR) and human epidermal growth factor receptors (Her-2). However TNBCs comprise a heterogeneous group of breast cancers and represents 10–20% of all breast cancer, with the majority expressing a basal-like phenotype [2]–[6]. Clinically, TNBCs behave more aggressively, with patients affected having a worse overall and disease-free survival when compared to other breast cancer subtypes. This has been partially attributed to the insensitivity of TNBCs towards available targeted treatment strategies, such as endocrine and anti-Her-2 therapies [7]–[8].

Nuclear factor kappa-B (NF-κB), a transcription factor, has been shown to be significantly increased in TNBC tumors, which is consistent with the aggressiveness of these tumors [9]. In the cytoplasm, NF-κB is bound to a group of inhibitory proteins known as inhibitors of NF-κB (IκB) [10]. The accumulation of non-phosphorylated IκB prohibits the translocation of NF-κB from the cytoplasm to nucleus, resulting in inactivation of NF-κB and its resultant downstream targets. NF-κB has been shown to promote the transcription of several key regulators of cancer invasion and progression, including cytokines, chemokines, cell adhesion molecules and inducible pro-inflammatory enzymes.

Additionally, NF-κB has been postulated to be a useful marker of epithelial-mesenchymal transformation (EMT) and invasiveness in breast cancers [11]–[12]. Thus, targeting genes induced by NF-κB activation, or inactivation of the NF-κB pathway, could serve as therapeutic targets for treatment of TNBC. EMT is one of the hallmarks of aggressive breast cancers and is associated with increased metastatic potential. EMT markers are overexpressed in TNBCs [13]. In particular FOXM1, which is an oncogenic transcription factor of the Forkhead family, has a well-defined role in cell proliferation and cell-cycle progression. Additionally, FOXM1 is over-expressed in breast cancer [14] and has been linked to EMT in pancreatic cancer [15].

Natural products have received increasing attention in recent years for utilization as novel anticancer agents [16]. Several natural compounds such as, withaferin A, honokiol, curcumin, quinones, plumbagin, *Phyllanthus watsonii,* cucurbitacin B and tanshinones, have been tested against breast cancer and revealed anticancer activity [17]–[24].

It has been known for many years that selected mushrooms of higher *Basidiomycetes* origin have anticancer properties [25]–[27]. Panepoxydone (PP), a compound isolated from *Lentinus crinitus* (an edible mushroom*)*, interferes with the NF-κB mediated signal transduction by inhibiting the phosphorylation of IκB [28]. Additionally, PP has been shown to inhibit tumor necrosis factor α (TNFα)-induced activation of NF-κB in COS-7 cells via inhibiting phosphorylation and degradation of IκB [28]. Furthermore, DNA microarray analysis of PP treated MonoMac6 cells showed decrease in the expression of thirty-three NF-κB-dependent pro-inflammatory genes without significant effects on the expression of house-keeping genes [29].

However, the role of PP against breast cancer is unexplored. Herein we report that PP has significant antitumor activity in breast cancer, with cell-line specific differential responses based upon tumor subtyping. For example, treatment with PP resulted in significant cytotoxicity, decreased invasion and migration, and increased apoptosis in all cell lines tested. Additionally, these changes correlated with changes in apoptosis-related protein expression, including up-regulation of Bax and cleaved PARP and down regulation of Bcl-2, survivin, cyclin D1 and caspase 3 in all breast cancer cell lines tested. However, there was difference in sensitivity of the cell lines to PP treatment, with resultant difference in their antitumor response, especially with the TNBC cells.

The antitumor effect of PP appeared to be related to its ability to inhibit the phosphorylation of IκBα, with cytoplasmic accumulation of NF-κB. PP treatment also down-regulated FOXM1, vimentin, zeb1, slug, and up regulated E-cadherin expression, which was similar to that observed after NF-κB silencing. These studies for the first time highlight the effect of PP on inhibiting aggressive breast cancers subtypes.

## Materials and Methods

### Drug and Reagents

Panepoxydone was procured from Alexis Biochemicals (San Diego, CA). Dimethyl sulfoxide (DMSO, vehicle control), Triton X-100, and bovine serum albumin (BSA) were obtained from Sigma-Aldrich (St. Louis, MO). Formaldehyde (16%) and 4',6-diamidino-2-phenylindole (DAPI) were purchased from Fisher Scientific (Suwanee, GA). Dulbecco's Modified Eagle Medium (DMEM), fetal-bovine serum (FBS), trypsin-EDTA, penicillin and streptomycin were purchased from Invitrogen (Carlsbad, CA).

For growth inhibition analysis, the CellTiter-Glo Assay was purchased from Promega (Madison, WI). Diff-Quick stain for invasion and migration analysis was purchased from Fisher Scientific (Newark, USA). PE Annexin V apoptosis detection kit I was obtained from BD Bioscience (San Diego,CA). For the translocation assay, the NF-κBp65 primary antibody was obtained from BD Transduction Laboratories (San Diego, CA) and the Alexaflour 488 immunofluorescence antibody was purchased from Invitrogen (Carlsbad, CA). siFOXM1 and siNF-kB was obtained from Santa Cruz Biotechnology (Santa Cruz, CA) and Cell Signaling Technology (Beverly, MA), respectively.

Primary antibodies against survivin, cyclin D1, poly (ADP-Ribose) polymerase (PARP), FOXM1, p21, CDK1, CDK2 and NF-kBp65 were purchased from Santa Cruz Biotechnology (Santa Cruz, CA) and Bcl-2, Bax, IkBα, pIκBα, caspase 3, cleaved PARP, E-cadherin, vimentin, zeb1,slug, cyclin E, cyclin B1 were procured from Cell Signaling Technology (Beverly, MA). Anti-rabbit, anti-mouse and anti-goat horseradish peroxidase-conjugated secondary antibodies were obtained from Santa Cruz Biotechnology (Santa Cruz, CA). The β-actin (mouse monoclonal) antibody was procured from Sigma-Aldrich (St. Louis, MO).

### Human breast cancer cell lines and culture conditions

The estrogen receptor positive MCF-7 and TNBC cells lines (MDA-MB-231, MDA-MB-468 and MDA-MB-453) were purchased from ATCC (Manassas, VA) and cultured in DMEM supplemented with 10% fetal bovine serum, penicillin (100 U/ml) and streptomycin (100 µg/ml) in a humidified 5% CO_2_ incubator at 37°C. Cells were sub-cultured biweekly with a split ratio of 1∶3. For treatments, stock solution of PP was prepared in DMSO (50 mM) and stored at −20°C in aliquots. At the time of experiments, dilutions were freshly prepared in complete growth medium. An equal volume of DMSO (final concentration, 0.2%) was added to the control.

### Cell proliferation assay

Breast cancer cells were seeded in 96-well plates at a density of 5×10^3^ cells/ well and after 18–20 hrs of incubation, cells were treated with PP or DMSO (0.2%, vehicle control) and incubation were continued for 72 hrs at 37°C. The inhibition of cell growth was determined using the luminescent CellTiter-Glo assay which measures viable cells based on adenosine triphosphate (ATP) content. Luminescence was measured using a VictorV (PerkinElmer, Waltham, MA) plate reader. GraphPad Prism 5 (GraphPad Software, Inc., La Jolla,CA) was used to construct graphs and calculate inhibitory concentration 50 (IC_50_) value.

### Cell cycle analysis

For cell cycle analysis cells were seeded in the 6 well plates with the density of 2×10^5^ cells per well, treated with different concentrations of PP and incubated at 37°C. After 24 hrs cells were fixed in methanol, stained with Popidium iodide/RNase binding buffer for 30 min at 37°C and analyzed by using flow cytometry on a BD-FACS CantoTM II (Becton-Dickinson, San Jose, CA) to calculate the percentage of cell population in various phases of cell cycle using Mod Fit LT software (Verity Software House, Topsham, ME).

### Cell Apoptosis Assay

Cells were seeded in the 6-well plates at a density of 1×10^6^ cells/well and after 24 hrs, treated with increasing concentrations of PP (based on IC_50_ values_)_ for 24 hrs. Cells were then harvested and stained using the PE Annexin V apoptosis detection kit to identify apoptotic cells according to the manufacturer's instructions followed by flow cytometry. This assay was used to quantify viable cells, early apoptotic cells and late apoptotic cells. Percentage of cell population in apoptosis was calculated using Mod Fit LT software (Verity Software House, Topsham, ME).

### Cell Migration/Invasion Assay

For *in-vitro* assessment of metastasis, migration and invasion assays were performed using a matrigel invasion chamber. The matrigel coated plates were rehydrated in warm DMEM serum-free medium for 2 hrs at 37°C. Cells in serum-starved media were seeded at the density of 5×10^4^ cells/well in 6-well inserts with 8 µm pore polycarbonate membranes for migration and in matrigel-coated inserts for invasion, and chemoattractant (DMEM with 10% FBS) was added in the plate chamber. Cells were incubated in 5% CO_2_ atmosphere at 37°C for 24 hrs. Non-invading cells were removed from the upper surface of the membrane by scraping using cotton swabs and cells which invaded through the matrigel to the bottom of the insert were fixed and stained with Diff-Quick cell staining kit and mounted on slide. Cells were observed under microscope and photographed using Nikon Eclipse TE 2000-U (Nikon Instruments Inc., Melville, NY). Ten random fields of view for each well were quantified by counting the cells in each field and averaging the results for each condition.

### siRNA transfection

siRNA targeting FOXM1and NF-kBp65 was used for the silencing of FOXM1 and NF-kBp65, respectively in MDA-MB-231 cells. Scrambled non-target siRNA was used as a negative control. For siRNA transfections, 2×10^5^ cells suspended in 2 ml of medium were seeded into a 6-well plate. After incubation for 24 hrs, cells were transfected with 50 nM siRNAs by using RNAiMax (Invitrogen, CA) according to the manufacturer's instructions. After 72 hrs proteins were collected and gene silencing efficiency was measured using immunoblotting. Expression of FOXM1 and EMT associated markers were checked on the silent proteins.

### Evaluation of Apoptosis, Cell cycle and EMT Related Protein Expression

Cells exposed to various concentrations of PP for 24 hrs were lysed and protein concentration was determined using DC protein assay kit (Biorad, Hercules, CA) following manufacturer's instructions. Total proteins (80 µg) in each cell lysate were subjected to resolution on 10% of sodium dodecyl sulfate polyacrylamide gel electrophoresis (SDS-PAGE) and electro-transferred onto polyvinylidene difluoride (PVDF) membranes. The membranes were incubated with blocking buffer (5% non-fat dry milk in phosphate-buffered saline) for 1 hour at room temperature (RT) and then further incubated with specific antibodies diluted in 5% non-fat dry milk overnight at 4°C. After washing with tris-buffered saline solution containing 0.1% Tween 20 (TBST), membranes were incubated with horseradish peroxidase-conjugated secondary antibodies for 2 hrs at RT followed by the washing with TBST. Blots were then treated with chemiluminescence reagents using a Super Signal West Femto Kit (Pierce, Rockford, IL) and the signal detected by using an LAS-3000 image analyzer (Fuji Photo Film Co., Tokyo, Japan). Each membrane was stripped and reprobed with anti-β-actin antibody to ensure equal protein loading. Densitometry was performed using an AlphaImager (Alpha Innotech Corp., San Leandro, CA).

### NF-kB Immunofluorescence Assay

MCF-7, MDA-MB-231, MDAMB-468 and MDAMB-453 cells (5×10^4^) were seeded in a 6-well plate and after overnight incubation at 37°C, treated with the top dose of PP (D3) as mentioned in Table 1 or same volume of 0.2% DMSO for 24 hrs. Cells were washed and fixed in 4% formaldehyde for 15 min at RT. The cells were then permeabilized with 1% Triton X-100 for 15 min at RT and blocked with 1% BSA for 30 min at RT. Cells were then incubated with NF-κBp65 antibody (1∶1000 in BSA) at 4°C overnight. After washing with PBS, the cells were incubated with the Alexaflour 488 antibody (1∶1000 in BSA) containing DAPI for 1 hour at 37°C. After washing, pictures were taken using the Nikon TE2000-U fluorescence microscope system (Nikon Instruments Inc., Melville, NY).

**Table 1:** Dose escalation of panepoxydone (PP) based on IC_50_ value.

Breast cancer cell lines	PP (µM) D1	PP (µM) D2	PP (µM) D3
MCF-7	2.5	5	10
MDAMB-453	2	4	8
MDAMB-468	3	6	12
MDAMB-231	7.5	15	30

### Statistical Analysis

All the experiments were performed at least twice independently and data presented as mean ± standard error mean. All data analysis was done using GraphPad Prism version 5.0 software. Statistical significance of difference was calculated using student's t-test with significant differences defined as at least a p value of <0.05.

## Results

### Anti-proliferative effect of PP in human breast cancer cells

To determine the effectiveness of PP, increasing concentrations of PP (0–50 µM) was exposed to MCF-7, MDA-MB-231, MDA-MB-468 and MDA-MB-453 cells and measured for inhibition of cell proliferation by CellTiter-Glo assay. PP exhibited a time and dose-dependent decrease in cell proliferation as early as 24 hrs and this continue to 72 hrs of exposure (Figure 1A), with IC_50_ values of 4, 5, 6 and 15 µM for MDA-MB-453, MCF-7, MDA-MB-468 and MDA-MB-231 cells, respectively (Figure 1B). Interestingly, MDA-MB-453 cells were the most sensitive, whereas the MDA-MB-231 was least sensitive to PP. Thus, for the reminder of experiments we utilized the half of IC_50_ values (D1), IC_50_ values (D2) and double IC_50_ values (D3) in the treatment of each cell line. Additionally, after PP treatment, morphologically, all cells appeared more rounded and many had become less adherent to the flask surface (Figure 1C).

**Figure 1:** Inhibitory effects of panepoxydone on the proliferation of human breast cancer cells. MCF-7, MDA-MB-231, MDA-MB-468 and MDA-MB-453 breast cancer cells were grown in 96 well microtitre plates (5000 cells/well) and treated with increasing concentrations of PP or with DMSO (0.2% vehicle control) and analyzed by CellTiter Glow assay. (**A**) Time-dependent anti-proliferative effect of PP on breast cancer cells. Data are presented as the means ± SD (n = 2). (**B**) Dose-dependent anti-proliferative effect of PP on breast cancer cells after 72 hrs. Data are presented as the means ± SD (n = 4). PP inhibited cell viability in a dose-dependent manner for all the cell types suggesting anti-cancer activity of PP. (**C**) Morphological changes of breast cancer cells after treatment with PP. Based on the IC_50_ value, 3 doses were selected for subsequent experiments: D1 (half of IC_50_, D2 (IC_50)_ and D3 (2×IC_50_). Cells (1.5×10^4^ cells/well) were seeded in 6-well plates and incubated with increasing concentrations of PP or DMSO (0.2% vehicle control) for 24 hrs. Morphological changes were observed under the inverted phase-contrast microscope and photographed. Representative micrographs are from one of the random fields of view (magnification 200X) of cells.

#### PP blocks cell cycle progression and modulates cell cycle regulatory proteins

We next asked if PP mediated growth suppression was due to its cell cycle intervention. To determine the effect of PP on the cell cycle alteration, all cell lines were evaluated by propidium iodide flow cytometry at 24 hrs. After PP treatment, MCF-7 cells showed 1.61 fold (10%–16.18%) whereas MDA-MB-468 revealed 2.52 fold (14.28%–35.94%) increase in G2 phase. Likewise MDA-MB-231 and MDA-MB-453 cells showed 1.76 fold (18.44%–32.58%) and 1.69 fold (19.99%–33.92%) increases in the S phase, respectively as compared to their individual controls (Figure 2A & 2B). Cell cycle checkpoints are important control mechanisms that ensure the proper execution of cell cycle events. Levels of cell cycle–regulated proteins were inhibited in all breast cancer cells. We found a dose-dependent decrease in the levels of CDK1, CDK2, cyclin B1 and cyclin E and increase in the p21 proteins. All these proteins are strongly associated with cell cycle arrest at G2/M and S phase (Figure 2C).

**Figure 2:** Effect of Panepoxydone on cell cycle phase distribution in breast cancer cells. (**A**) MCF-7, MDAMB-231, MDAMB-468 and MDAMB-453 breast cancer cells (2×10^5^ cells/well) were seeded in 6 well plates, treated with PP or DMSO (0.2%, vehicle control) for 24 hrs and subsequently stained with propidium iodide (PI) followed by flow cytometry. The left triangle crest is the G1 phase, the right crest is the G2/M phase, and the middle area is the S-phase. Data are representative of one of the two independent experiments. (**B**) Histogram constructed on the mean value of two independent experiments. MCF-7 and MDAMB-468 cells accumulated in G2-phase whereas increase in S-phase was observed for MDAMB-231 and MDAMB-453 cells after PP treatment. (**C**) Total protein was isolated from control and PP-treated breast cancer cells and subjected to immunoblotting of p27, CDK1, CDK2,cyclin B and cyclin E proteins. Membranes were stripped and re-probed with anti-actin antibody to ensure equal protein loading. This data indicate the possible role of PP in inducing cell cycle arrest at G2 and S phase.

### PP induces apoptosis and increased cell survival proteins

Next we sought to determine if PP induces apoptosis. Apoptosis was quantitatively measured using the PE Annexin V staining flow cytometry method. PP treatment resulted in a significant increase in the number of apoptotic cells in all breast cancer cell lines, but to varying degrees (Figure 3A). Interestingly, highest dose (10 uM) of PP in MCF-7 cells showed a relatively low percentage of apoptotic cells (1.2 fold), as compared to MDA-MB-231 (2 fold), MDAMB-468 (2.9 fold) and MDA-MB-453 (5.2 fold) when compared with their respective controls (Figure 3B).

**Figure 3:** Panepoxydone induces apoptosis in breast cancer cells. (**A**) MCF-7, MDA-MB-231, MDA-MB-468 and MDA-MB-453 breast cancer cells were grown in a 6-well plate (1×10^6^ cells/well) and treated with increasing concentrations of PP or DMSO (0.2% vehicle control) for 24 hrs. After treatment, cells were stained with 7-AAD and PE Annexin V followed by flow cytometry. Unstained DMSO-treated cells served as a negative control. Data show a dose-dependent increase in the number of apoptotic cells in all breast cancer cells after treatment with PP as compared to control cells. A representative picture of two independent experiments is shown. (**B**) Histogram representation of increased number of apoptotic cells in breast cancer cells after treatment with PP. (**C**) Total protein was isolated from control and PP-treated breast cancer cells and subjected to immunoblotting of apoptosis an dsurvival related proteins. Membranes were stripped and re-probed with anti-actin antibody to ensure equal protein loading. Bax and cleaved PARP was upregulated and Bcl-2, survivin, cyclin D1 and caspase 3 was down-regulated in all breast cancer cells in a dose-dependent manner. (**D**) Bar diagram indicate the increased Bax/Bcl-2 ratio in all breast cancer cells after PP treatment indicating its role in apoptosis. * indicates statistically significant difference between PP treated and untreated cells at p<0.05 (*), p<0.01(**), and, p<.001(***) levels by student's t-test. Altogether this data indicate the possible role of PP in modulation of apoptosis related genes. Immunoblotting for each protein was performed at least twice.

Bax and Bcl-2 belong to a multi-gene family of proteins that play an important role in the regulation of apoptosis. Bcl-2 is anti-apoptotic protein and promotes cell survival, whereas Bax is pro-apoptotic protein and antagonizes the effect of Bcl-2 [30]. Following PP treatment, in all the cell lines there was an increase in Bax expression, with concomitant decrease in Bcl-2 protein expression, which is consistent with increased apoptosis (Figure 3B & 3C). Furthermore, the ratio of Bax/Bcl2, a commonly used measure of overall apoptosis effect, was significantly increased in all the TNBC cell lines. The ratio of Bax/Bcl2 was highest for the MDAMB-453 (32 folds) (Figure 3D).

To confirm that PP induces apoptosis, we assayed both cyclin D1, survivin, and caspase expression at the protein level in the presence of PP. Cyclin D1 and survivin both were down-regulated (2–7.5 folds) in a dose-dependent manner as demonstrated by western blot, in all breast cancer cell lines after PP treatment (Figure 3C). Caspase 3 expression was decreased in all TNBC cell lines; with the exception of MCF-7 cells, which are caspase 3 deficient [31]. Treatment with PP also triggered PARP cleavage (2-4 folds) in the TNBC cells lines. In the absence of caspase 3, no cleaved PARP was detected in MCF-7 cells (Fig 3C).

### PP inhibits NF-κB activation and translocation

NF-κB is normally localized in the cytoplasm in an inactivate form and bound to non-phophorylated IκBα. During activation, IκB is phosphorylated and thus disassociates from NF-κB. This then allows NF-κB to translocate from the cytoplasm to the nucleus where it then regulates the expression of several genes. The effect of PP on the expression of IκBα and its phosphorylated form (pIκBα) was evaluated by western blot. Figure 4A reveals that there was a dose-dependent down-regulation of pIκBα, with concomitant up-regulation of IκBα, in response to PP treatment in all the cell lines tested.

**Figure 4:** Panepoxydone inhibited NF-kB: (**A**) Immunoblotting of IkB and pIkBα showed accumulation of IkBα (inactive) and down-regulation of pIkBα (active) in PP treated breast cancer cells. This indicates the potential of PP in keeping NF-kB in the active state. (**B**) Bar diagram indicate the increased IkB/pIkB ratio in all breast cancer cells after PP treatment. * indicates statistically significant difference between PP treated and untreated cells at p<0.05 (*), p<0.01(**), and, p<.001(***) levels by student's t-test. (**C**) Localization of NF-κB was done on MCF-7, MDAMB-231, MDAMB-468 and MDAMB-453 breast cancer cells that were fixed, permeabilized and labeled with anti-p65 subunit of NF-κB then nuclei were stained with DAPI. Controls cells were compared to cells treated with the top dose of PP (D3). Controls cells showed increased expression of NF- κB in the nucleus, whereas following treatment with PP, NF-κB accumulated in the cytoplasm, indicating decreased activity.

Again, differences between MCF-7 and the TNBC cell lines were noted. When the ratio of pIκBα/IκBα was calculated, there was at least a two-fold difference between the MCF-7 cell line and the TNBC cells as a whole. Furthermore, again the MDA-MB-453 cells appeared to be more sensitive to PP, with the ratio of pIκBα/IκBα highest in this group (up to 7-folds) following PP treatment (Figure 4B).

To determine if the resultant increase in non-phosphorylated IκBα results in a decreased translocation of NF-κB from the cytoplasm to nucleus, we performed an immunofluorescence assay for the localization of NF-κB following PP treatment. Visualization of cells after PP treatment showed reduced expression of NF-kB in the nucleus in all the cell lines evaluated (Figure 4C).

### PP reduces cell migration and invasion

NF-kB is well recognized to be a multi-functional protein involved not only in the regulation of cell proliferation, but in cell migration and invasion as well [32]. Since numerous reports have demonstrated that PP targets NF-κB, we next sought to determine the effect of PP on the migratory and invasiveness of TNBC cells. Migration (Figure 5A) and invasion (Figure 5B) of breast cancer cells was evaluated by using noncoated and matrigel-coated chambers, respectively. A dose-dependent decrease in migration and invasion was noted in all of the cell lines following treatment with increasing concentrations of PP. Cell-line specific sensitivity to PP was noted between MCF-7 and the TNBC cells, with significant decrease in migration and invasion noted only at the highest dose of PP in MCF-7 cells.

**Figure 5:** Panepoxydone decreases migration and invasion properties of breast cancer cells. MCF-7, MDA-MB-231, MDA-MB-468 and MDA-MB-453 cells were seeded on noncoated or matrigel-coated membranes for motility (**A**) and invasion (**B**) assays, respectively and incubated for 24 hrs. DMEM containing 10% fetal bovine serum in the lower chamber was used as a chemoattractant. After incubation, cells that had migrated or invaded through the membrane/matrigel to the bottom of the insert were washed, fixed, stained and counted in ten random microscopic fields. The histograms show mean of two independent experiments and the error bar represent SEM. * indicates statistically significant difference between PP treated and untreated cells at p<0.05 (*), p<0.01(**), and, p<.001(***) levels by student's t-test. Results indicate reduction in the migrated and invaded cells after PP treatment in a dose dependent manner.

Furthermore, although general cytotoxicity to PP in MCF-7 cells was close to that of its counterpart, the luminal- type triple negative MDA-MB-453 cells (Figure 1C), breast cancer subtype-associated differences were noted with regard to migration and invasion (Figure 5A, 5B). For example, there was a marked difference in the effect of PP on migration and invasion capabilities of MCF-7 cells when compared to MDA-MB-453 at the highest dose tested (1.72 vs 3.95/1.82 vs 2.77-folds over control), which correlates to the aggressiveness in TNBCs.

### PP causes EMT reversal through FOXM1

Studies have shown that down-regulation of FOXM1 in breast cancer cells by RNA interference led to inhibition of proliferation, migration and invasion of cancer cells [33].

Using in silco analysis we determined that the FOXM1 promoter has a binding site for NF-kB. Thus, we were interested to examine the relationship between FOXM1 and NF-κB.

PP treatment significantly reduced FOXM1 expression in MCF-7 and MDA-MB-231 (1.7 and 2.4-fold, respectively, p<0.05) but not in MDAMB-453 and MDAMB-468 cells when analyzed through western blot analysis. The effect of PP on decreasing FOXM1 expression was comparable to si-NFNF-kB treatment in MDAMB-231 cells (Figure 6A).

**Figure 6:** Panepoxydone modulates EMT related markers. Total protein was isolated from control and PP-treated breast cancer cells and subjected to immunoblotting of proteins. Membranes were stripped and re-probed with anti-actin antibody to ensure equal protein loading. (**A**) Immunoblotting of FOXM1 after PP treatment and silencing of FOXM1 and NF-κB. (**B**) Immunoblots of cell lysates treated with PP or silenced FOXM1 and NF-kB for E cadherin, vimentin, slug and zeb-1. (**C**) Bar diagram indicate the fold difference in the EMT markers after PP treatment and above specified silencing. * indicates statistically significant difference between PP treated and untreated cells at p<0.05 (*) and p<0.01(**) levels by student's t-test. Altogether this data indicate the PP induced EMT reversal is through FOXM1 in breast cancer cells.

Furthermore, we identified that treatment with PP resulted in alteration of EMT-associated proteins with a significant increase in epithelial marker, E-cadherin (1.8 to 4.2-fold, p<0.05) and a decrease in mesenchymal markers, vimentin, slug and zeb1 in the MDA-MB-231 cells (1.5–4.2 fold, p<0.05). To further elucidate the relationship between FOXM1 on EMT reversal, we then silenced FOXM1 and NF-kB in MDA-MB-231 cells and evaluated its effect on the EMT-associated markers. Again we noted up-regulation of E cadherin (3.5-fold, p<0.01) and down-regulation of vimentin, slug and zeb1 (4.fold, p<0.01) (EMT reversal) in si-FOXM1 and si-NF-kB treated cells, which was similar to what we observed in the PP-treated MDA-MB-231 cells (Figure 6B & 6C).

## Discussion

Breast cancer is the leading cause of cancer in women world-wide [1].

Based on gene expression profiling, breast cancer have been classified into four main subtypes - luminal A, luminal B, Her-2+ enriched and basal-like. This classification is used to direct the use of targeted therapies such as endocrine-based therapy for hormone receptor positive (HR+) breast cancer and Her2-based therapy such as trastuzumab, lapatinib and pertuzumab for Her2-enriched cancers [34]–[35]. The use of this molecular-based approach in the treatment of breast cancer has revolutionized how we treat breast cancer in the last several decades and is the main contributor to the decreased mortality noted.

However, approximately 20% of all breast cancers are diagnosed as TNBC. Because TNBC lacks all three of the molecular targets such as ER, PR and Her2, it cannot be treated with currently available targeted therapies such as hormone therapies or Her2-based therapies. Furthermore, since the genes linked to TNBCs are not well understood at this time, targeted therapies directed to TNBC do not yet exist. Therefore, TNBC is usually treated with some combination of surgery, radiation therapy and chemotherapy. Thus, due to aggressive nature of this disease, and with few treatment options and no targeted therapies specifically for TNBC, a continuous search for better treatment options is warranted.

Traditionally, the term TNBC has been used synonymously with basal-like breast cancer. Most TNBCs are basal-like and most basal-like tumors are triple negative. However, not all TNBCs are basal-like and not all basal-like tumors are triple negative. In fact, recently, TNBCs have been classified into 6 subclasses based upon the presence of unique gene expression profiles. These include two basal-like (BL1 and BL2), an immunomodulatory (IM), a mesenchymal (M), a mesenchymal stem–like (MSL), and a luminal androgen receptor (LAR) subtype [36]. It is expected that selection of TNBC tumor subtypes will be helpful in the development of targeted agents and also serve as a key model for preclinical studies. Additionally, it is expected that this information would be useful to further identify biomarkers that can be used for patient selection in the design of clinical trials for TNBC, as well as to monitor their response to treatment.

NF-κB has been shown to have increased expression in TNBC tumors and may account for the aggressiveness of these tumors. It is well known that NF-κB plays a significant role in many signaling pathways including those that are involved in cancer development and progression [37]. For example, NF-κB promotes the transcription of several cytokines (e. g. TNF-α, IL-1β, IL-6, IL-2), chemokines (IL-8), macrophage inflammatory protein-1 α (MIP-1α), cell adhesion molecules (e. g. E-selectin, ICAM-1, VCAM-1) and inducible pro-inflammatory enzymes like NO synthase II and cyclooxygenase-2 [38]. Furthermore, increased NF-κB activity is associated with enhanced cancer cell survival, by inhibiting apoptosis in breast and pancreatic cancer [39]-[40], through transcriptional regulation of anti-apoptotic proteins (IAPs, FLIP, and Bcl-XL) and cyclin D1 [41]. Thus, it's reasonable to assume that inhibition of the NF-κB pathway and its target genes, could serve as a therapeutic target for the treatment of TNBC.

Although several synthetically derived NF-kB inhibitors have been proposed [42], there are few studies that have investigated the effect of natural compounds on NF-kB expression and/or translocalization. Panepoxydone (PP), which is isolated as a secondary metabolite from Basidiomycetes (*Lentinus crinitus)*, was first identified as an important regulator of inflammation, autoimmune diseases and apoptosis [29] and was subsequently found to be a natural NF-κB inhibitor [28]–[29]. However, there are only a limited number of reports investigating the effect of this natural metabolite in cancer, and none to our knowledge in breast cancer.

Our results indicate that PP has significant anti-tumor activity against all breast cancer cells in a dose- and time-dependent manner with MDA-MB-453 cells demonstrating the most sensitivity and lowest IC_50_ value. Indeed, the effect of PP appears to be mediated though NF-kB, as we observed nuclear to cytoplasmic translocation shift, which coincides with decreased pIkB expression and increased total IkB expression in all cell lines, which is responsible for release of NF-κB from the cytoplasm where it can then be transported into the nucleus [43].

Several reports have shown that nuclear localization (activation) of NF-κB and the expression of Bcl-2 serve as an important component for resistance to therapy in human cancers [44]–[47]. A key determinant in the apoptotic process is the balance of anti-and pro-apoptotic proteins with an increased ratio of pro-apoptotic proteins (Bax and Bim) to anti-apoptotic proteins (Bcl-2 and Bcl-xL) leading to apoptosis and eventually cell death. PP significantly decreased Bcl-2 expression and increased Bax expression in all cell lines, with overall net increase in the Bax/Bcl-2 ratio, with MDA-MB-453 cells demonstrating significantly higher ratios. These results were corroborated with flow cytometry analysis of Annexin V staining, and subsequent PARP cleavage through activation of increased caspase 3 expression, which are well established indicators of apoptosis. Thus, it is plausible that PP's inhibitory effect is mediated through the Bcl-2 pathway.

Cyclin D1 is one of the most commonly overexpressed proteins in breast tumors and involved in regulation of transition from the G1 to S phase during the cell cycle [48]. Furthermore, a high level of survivin expression is associated with poorer patient prognosis in breast carcinoma [49]–[50]. Survivin, a member of the inhibitor of apoptosis (IAP) family is highly expressed in most human tumors including breast cancer and plays a critical role in both control of cell division and inhibition of apoptosis [51]–[53]. PP treatment resulted in decreased expression of cyclinD1 and survivin. Collectively, these results show the mechanisms by which PP is exerting its anti-tumor affect, specifically via modulation of apoptotic-related proteins and modulation of DNA repair via PARP cleavage. More importantly, it emphasizes the ability of a targeted therapy, such as an NF-κB inhibitor, to trigger a diverse cascade of events that can lead to breast cancer cell death, particularly in the luminal A subtype of TNBC.

Tumor cell migration and invasion are key steps in the development of metastasis and play a significant role during the process of distant metastasis [54]. TNBC cells are considered more aggressive than other breast cancer cells and are characterized by increased migration and invasion capabilities. Our results demonstrate that treatment with PP has a direct effect on aggressive features of breast tumors, such as cell migration and invasion, however as with the cytotoxicity experiments, there is differing effectiveness in the cell lines. For example, although MCF-7 cells and MDAMB-468 and MDA-MB-453 cells shared very close IC_50_ values, PP treatment differed with regard to inhibiting their invasion capability. A significant reduction in the migration and invasion was observed at IC_50_ dose (dose D2) in all the TNBC cells lines; however, it was not significant for the MCF-7 cells. The fact that both MCF-7 and MDA-MB-453 cell lines showed similar IC_50_ values compared to the other TNBC cell lines, but demonstrated a different inhibitory effect on the migratory and invasion capability, further highlights that PP is most effect in luminal type tumors. This is not surprising, since TNBC cells (MDA-MB-453, luminal type) are more aggressive in nature as compared to ER positive (MCF-7) cells.

The fact that PP was able to have a significant general effect on cytotoxicity in all the breast cancer cell lines, but also exhibit cell-line specific effects on critical features associated with the aggressiveness of TNBC is of extreme importance. It highlights the role of utilizing therapeutic agents to help in elucidating the underlying mechanisms involved in specific tumor biology, prior to clinical translation. The pattern of anti-tumor activity of PP (MDA-MB-453 > MDA-MB-468 > MDA-MB-231) in all three TNBC cell lines is similar to that reported for 17-dimethylaminoethylamino-17-demethoxygeldanamycin (17-DMAG), a heat shock protein (Hsp90) inhibitor [35]. Hsp90 has been identified as a critical and multimodal target for the treatment of TNBC. Reports have already shown the significance of Hsp90 inhibitors (PF-4942847, PU-H71) for the development of targeted therapies against TNBC [55]–[56] and an interesting future study would be to determine the effect of PP onHsp90 expression.

An essential feature of metastasis is an epithelial to mesenchymal transition (EMT) or loss of E-cadherin expression [57]–[58]. This allows for increased cell migration, local or distant invasion. The TNBC cell culture models, MDA-MB-468, MDA-MB-453, and MDA-MB-231 [36], are all highly migratory and have the mesenchymal phenotype. FoxM1 is known to be a key regulator of transition from G1 to S phase as well as for the progression to mitosis [59]–[60], Members of the FOXM1 family involved in the development and progression of breast, liver, prostate, brain, and lung cancers through their ability in driving cell cycle progression and evasion of growth arrest [61]. FOXM1 expression has been shown to correlate with increased proliferation in prostate and lung cancer [62]–[63]. In breast cancer FOXM1 down-regulation leads to inhibition of proliferation, migration and invasion of breast cancer cells indicating the new approach for treatment of breast cancer [33].

We found that treatment with PP caused a down-regulation of FOXM1. Interestingly, silencing NF-kB reduces the expression of FOXM1, similarly to PP treatment, which is concomitant to upregulation of E-cadherin expression and down regulation of (vimentin, slug and zeb1). Thus, our results indicate the potential of PP in down-regulating FOXM1 and well established mesenchymal markers as well as induce the expression of epithelial marker, E-cadherin in breast cancer cells. Altogether these results highlight that the PP induced EMT reversal is through inhibition of FOXM1 in breast cancer cells (Figure 7).

**Figure 7:** Schematic diagram of PP-induced cell death mechanism and EMT reversal.

A recent report indicated that FOXM1 promotes EMT in breast cancer cells by stimulating the transcription of EMT-related genes and metastasis of breast cancer cells in vivo [64]–[65]. In silco analysis of the FOXM1 promoter revealed the presence of NF-kB binding sites. The fact that PP decreases FOXM1 possibly through inhibition of NF-kB activity further strengthens the rationale that targeting NF-kB is a rationale clinical approach to treat breast tumors, particularly TNBC.

## Conclusions

In summary, our results demonstrate that targeting NF-kB with PP can have significant anti-tumor activity against breast cancer cells, through inhibition of cell growth, and a reversal of EMT. Furthermore, our observation that PP has cell line specific differences in the TNBC cell lines, highlights the need to employ a more rational and evidence-based approach in evaluation of novel therapeutic agents in the treatment of cancer. Given the recent sub-classification of TNBC, and our findings that cell lines representing different subtypes of TNBC have varying responses to PP, supports the contention that not all TNBC should be treated the same. In fact, these findings correlate well with clinical findings observed in the treatment of patients with TNBC; with many patients having chemotherapy-sensitive associated with a complete pathological responses and thus a favor outcome. However, other TNBC patients tend to have very aggressive disease with very poor prognosis. At this point, we have not yet been able to preselect which patients may response to chemotherapy.

Thus, these results highlight the need for a more evidence-based selection of therapies in patients with TNBC to achieve optimal response. Use of targeted therapies, such as PP, can not only help further characterize the molecular processes involved in the aggressiveness of this disease, but also provide a rational approach to discover potential new targets for the treatment of TNBC.

A limitation to this study is that these are only *in-vitro* experiments. Further studies will be required to check the effect of PP on healthy breast cancer cells and also appropriate *in-vivo* models. These additional studies are required to establish PP as a therapeutic agent for the treatment of triple negative breast cancer.
